The article "Abnormal Mitochondria-Endoplasmic Reticulum Communication Promotes Myocardial Infarction" was retracted in 2022. Reasons: compromised peer review; original data or images not available; unreliable data.

# Abnormal Mitochondria-Endoplasmic Reticulum Communication Promotes Myocardial Infarction

**DOI:** 10.3389/fphys.2021.717187

**Published:** 2021-08-03

**Authors:** Degang Cheng, Jia Zheng, Fang Hu, Wei Lv, Chengzhi Lu

**Affiliations:** Department of Cardiology, Tianjin First Central Hospital, Tianjin, China

**Keywords:** mitochondria-endoplasmic reticulum communication, BAP31, FIS1, myocardial infarction, cell death

## Abstract

Myocardial infarction is characterized by cardiomyocyte death, and can be exacerbated by mitochondrial damage and endoplasmic reticulum injury. In the present study, we investigated whether communication between mitochondria and the endoplasmic reticulum contributes to cardiomyocyte death after myocardial infarction. Our data demonstrated that hypoxia treatment (mimicking myocardial infarction) promoted cardiomyocyte death by inducing the c-Jun N-terminal kinase (JNK) pathway. The activation of JNK under hypoxic conditions was dependent on overproduction of mitochondrial reactive oxygen species (mtROS) in cardiomyocytes, and mitochondrial division was identified as the upstream inducer of mtROS overproduction. Silencing mitochondrial division activators, such as B cell receptor associated protein 31 (*BAP31*) and mitochondrial fission 1 (*Fis1*), repressed mitochondrial division, thereby inhibiting mtROS overproduction and preventing JNK-induced cardiomyocyte death under hypoxic conditions. These data revealed that a novel death-inducing mechanism involving the BAP31/Fis1/mtROS/JNK axis promotes hypoxia-induced cardiomyocyte damage. Considering that BAP31 is localized within the endoplasmic reticulum and Fis1 is localized in mitochondria, abnormal mitochondria-endoplasmic reticulum communication may be a useful therapeutic target after myocardial infarction.

## Introduction

Mitochondria-dependent cardiomyocyte death is one of the primary pathogenic contributors to myocardial infarction (Heusch, 2019; Zhu et al., 2021). In clinical practice, thrombolytic therapy and/or percutaneous coronary interaction surgery are the standard methods of enhancing cardiomyocyte survival in patients with myocardial infarction (Gori et al., 2020; Kleinbongard, 2020; Watson et al., 2020). Despite advances in the treatment of myocardial infarction, the molecular pathways underlying ischemia-induced cardiomyocyte death are not fully understood (Wang et al., 2020b,c; Wang and Zhou, 2020; Zhu and Zhou, 2021). Determining the upstream signals of mitochondria-dependent cardiomyocyte death will enable the development of therapeutic approaches to improve cardiomyocyte survival during or after myocardial infarction (Hillmeister et al., 2020; Pflüger-Müller et al., 2020).

The article "Abnormal Mitochondria-Endoplasmic Reticulum Communication Promotes Myocardial Infarction" was retracted in 2022. Reasons: compromised peer review; original data or images not available; unreliable data.

Mitochondria-dependent cell death is primarily executed by c-Jun N-terminal kinase (JNK), which translocates to the nucleus to upregulate pro-apoptotic genes upon certain stimuli (Javadov et al., 2014). Impaired mitochondrial structure or function due to oxidative stress, energy depletion, mitochondrial membrane damage or mitochondrial DNA injury can induce the JNK pathway. In addition, stress-related proteins such as Macrophage stimulating 1 (Wang and Song, 2018), BCL2 interacting protein 3 (Li et al., 2018) and protein kinase C epsilon/delta (Nuñez et al., 2017) have been found to activate the JNK pathway. Among these various stimulants, mitochondrial oxidative stress seems to be the main inducer of JNK (Larson-Casey et al., 2020; Seano and Jain, 2020). Interestingly, JNK pathway activation has been reported to exacerbate cardiomyocyte oxidative stress by inducing mitochondrial reactive oxygen species (mtROS) overproduction (Jin et al., 2018). Activated JNK inhibits the activity of mitochondrial anti-oxidative enzymes such as superoxide dismutase 2 (SOD2) (Liu et al., 2020). JNK pathway activation has also been associated with increased nuclear factor κB activity, which accelerates mtROS generation by suppressing the mitochondrial respiratory complexes (Mu et al., 2020). This positive feedback between mtROS and JNK amplifies the damage signals to mitochondria and irreversibly impairs their function and structure, creating the early conditions for mitochondria-dependent cell death (Unterleuthner et al., 2020; Watson et al., 2020).

Although the relationship between mtROS and JNK has been carefully illustrated, the upstream activators of these molecules remain to be fully characterized (Hamilton et al., 2020; Lahiri et al., 2020). Recently, mitochondrial division was reported to promote mtROS overproduction (Tan et al., 2020; Wang et al., 2020a). Excessive mitochondrial division fosters the uneven distribution of mitochondrial DNA into daughter mitochondria, thus increasing the amount of broken mitochondrial DNA (Wang et al., 2020e,f). Damaged mitochondrial DNA then fails to synthesize the mitochondrial respiratory complexes, so mitochondrial oxidative phosphorylation is repressed and mtROS are overproduced (Zhou et al., 2018a; Wang et al., 2020d).

Mitochondrial division depends on the cooperation between mitochondrial fission factors and the endoplasmic reticulum (ER) (Chang et al., 2021; Zhu and Zhou, 2021). The ER provides anchoring strength to promote mitochondrial contraction, while mitochondrial fission factors such as mitochondrial fission 1 (Fis1), dynamin-related protein 1 (Drp1), mitochondrial fission factor (Mff), mitochondrial dynamics protein of 49 kDa (Mid49) and mitochondrial dynamics protein of 51 kDa (Mid51) perform the contraction (Zhou et al., 2018b; Lobo-Gonzalez et al., 2020). Among these proteins, Fis1 is thought to contribute to myocardial infarction (Cheng et al., 2020), as Mdivi-1 treatment significantly reduced the infarcted area by preventing Fis1 from binding to Drp1 (Jannuzzi et al., 2020; Li et al., 2020). Recently, the binding between mitochondria-localized Fis1 and ER-expressed B cell receptor associated protein 31 (BAP31) was reported to stimulate mitochondria-dependent apoptosis by bridging the mitochondria-ER interface (Iwasawa et al., 2011). Thus, in this study, we asked whether interrupting the cooperation between BAP31 and Fis1 could inhibit mtROS/JNK-induced cardiomyocyte death in order to treat myocardial infarction.

The article "Abnormal Mitochondria-Endoplasmic Reticulum Communication Promotes Myocardial Infarction" was retracted in 2022. Reasons: compromised peer review; original data or images not available; unreliable data.

## Materials and Methods

### Cell Culture and Treatment

H9c2 cardiomyocytes derived from the rat myocardium were purchased from the American Type Culture Collection cell bank. The cells were cultured in Dulbecco’s modified Eagle’s medium containing 10% fetal bovine serum, 100 IU/L penicillin and 100 μg/mL streptomycin in a 37°C incubator containing 95% air and 5% CO_2_. When the cells were 90% confluent, the culture medium was substituted with starvation medium (Dulbecco’s modified Eagle’s medium without fetal bovine serum) for 24 h (Detter et al., 2020). Then, the starvation medium was replaced with pre-anoxic sugar-free D-Hank’s solution and drug solutions (high, medium or low concentrations of Kaji-ichigoside F1, or Verapamil as a positive control). Kaji-ichigoside F1 and Verapamil were purchased from Wuhu Delta Medical Technology Co., Ltd. (purity > 99%; Anhui, China) (Mossoba et al., 2020).

### Hypoxia/Reoxygenation

Cardiomyocytes were cultured in hypoxic medium with a mixed gas consisting of 95% N_2_ and 5% CO_2_ at 37°C for 24 h, and then were cultured in fresh culture medium with a mixed gas consisting of 95% air and 5% CO_2_ for 12 h (Singh et al., 2020). The cells in the control group were cultured under normal conditions with 95% O_2_/5% CO_2_ at 37°C (Zhou et al., 2019).

### Anti-oxidative Enzyme Evaluation

Cardiomyocytes were collected and centrifuged at 3,000 × *g* for 10 min at 4°C. The supernatants were collected, and GSH, SOD, and GPX levels were detected using commercial kits according to the manufacturer’s instructions (Beyotime Biotechnology, Shanghai, China) (Ollauri-Ibáñez et al., 2020).

### Transfection

Twenty-four hours before transfection, H9c2 cells were seeded in six-well plates (2 × 10^5^ cells per well) and incubated overnight. Then, the cells were transfected with a control vector or with siRNAs against *Fis1* or *BAP31* using Lipofectamine 3000 reagent (Invitrogen Life Technologies, United States) and Opti-MEM medium (Invitrogen Life Technologies) in accordance with the manufacturer’s specifications (Szaraz et al., 2020). The siRNAs were purchased from Tolo Biotech (Shanghai, China).

The article "Abnormal Mitochondria-Endoplasmic Reticulum Communication Promotes Myocardial Infarction" was retracted in 2022. Reasons: compromised peer review; original data or images not available; unreliable data.

### ROS Evaluation

After treatment, cardiomyocytes were incubated with 2,7-dichlorofluorescein diacetate (Jiancheng, Nanjing, China) at 37°C for 40 min. The mean fluorescence intensity was detected using an automatic fluorescence microplate reader (Bio-Rad, United States) (Shi et al., 2018).

### Detection of Mitochondrial Membrane Potential

A JC-1 mitochondrial membrane potential assay kit (Beyotime Biotechnology) was used to detect the mitochondrial membrane potential in H9c2 cells. Cold phosphate-buffered saline was used to wash the cells after the hypoxia treatment (Islam, 2020). Then, 1 mL of cell culture medium and 1 mL of JC staining working fluid were added, and the cells were incubated for 30 min. Subsequently, the cells were washed twice with JC-1 staining buffer. The cells were observed using fluorescence microscopy, and changes in the mitochondrial membrane potential were determined based on changes in the fluorescence intensity at different excitation and emission wavelengths. JC-1 aggregates were observed at a maximum excitation wavelength of 585 nm and a maximum emission wavelength of 590 nm, while JC-1 monomers were observed at a maximum excitation wavelength of 514 nm and a maximum emission wavelength of 529 nm (Ednie and Bennett, 2020).

### Cell Viability

Cells were cultured on a 96-well plate and transfected with siRNAs or mimics for various times. Then, 24–48 h after transfection, the cells were seeded into 96-well plates (3000 cells per well), and cell viability was measured using a CCK-8 assay (Beyotime) according to the manufacturer’s instructions (Umapathy et al., 2020). The absorbance was detected on a microplate reader at 450 nm. The experiments were performed at least three times (Heimerl et al., 2020).

### Western Blotting Analysis

Cells were harvested and boiled in lysis buffer containing protease inhibitors. The total protein lysates were electrophoretically separated on 10% sodium dodecyl sulfate polyacrylamide gels and transferred to polyvinylidene difluoride membranes (Millipore) (Bausch et al., 2020). Then, the membranes were blocked with 5% skim milk for 3–4 h at room temperature and incubated with primary antibodies (1:1,000) at 4°C overnight (Lu et al., 2020). The membranes were subsequently washed with Tris-buffered saline containing Tween 20 and incubated with an appropriate horseradish peroxidase-conjugated secondary antibody (1:5,000) at room temperature for 1 h. Enhanced chemiluminescence was used to detect the results.

The article "Abnormal Mitochondria-Endoplasmic Reticulum Communication Promotes Myocardial Infarction" was retracted in 2022. Reasons: compromised peer review; original data or images not available; unreliable data.

### ELISA

Cells were centrifuged at 2,000 rpm for 15 min, and their supernatants were collected. Then, inflammatory factors [interleukin (IL)-8, IL-6, TNF-α and IL-10] in the cell supernatants were measured using ELISA kits (Nanjing Jiancheng Institute of Biological Engineering) in strict accordance with the kit instructions (Qiao et al., 2020; Selvaraju et al., 2020).

### Apoptosis Assay

Cells were fixed with 4% paraformaldehyde at room temperature for 1 h, and then were treated with 0.5% Triton X-100 for 1 h. The cells were washed twice with phosphate-buffered saline, and then apoptosis was analyzed with a TUNEL Apoptosis Assay Kit (Beyotime Biotechnology) in strict accordance with the manufacturer’s instructions (Santosa et al., 2020). Finally, the nuclei were stained with 0.5 g/mL 4′,6-diamidino-2-phenylindole for 4 min (Schinner et al., 2020). Apoptotic cells (those with nuclei dyed brown-yellow) were observed and photographed under a fluorescence microscope.

### RNA Extraction and cDNA Synthesis

Total RNA was extracted from frozen tissues and cells (HT-29 cell line and colorectal CSC-enriched spheroids) using an miRNeasy mini kit (QIAGEN GmbH, Germany) according to the manufacturer’s instructions (Pabel et al., 2020). RNA samples were separated using agarose gel electrophoresis, and the RNA concentration was measured based on the optical absorbance at 260/280 nm (Wincewicz and Woltanowski, 2020). Then, cDNA was synthesized from the extracted RNA using a cDNA synthesis kit (TaKaRa Bio, Shiga, Japan) and an miRNA cDNA synthesis kit (Bon Yakhteh, Iran).

### qRT-PCR

Specific primers for qRT-PCR were designed using Primer-BLAST (65) and OligoAnalyzer 3.1 software (Integrated DNA Technologies) (Zhu et al., 2018). Then, qRT-PCR was performed using SYBR Green PCR Master Mix (TaKaRa) on a Real-Time PCR System (Rotor-Gene Q MDx, Germany). The levels of miRNAs and *TPTEP1* were normalized to those of the internal control of the kit and *RNU6* (*U6*), respectively (Le Cras et al., 2020). *GAPDH* was used as an internal control to normalize the expression of other mRNAs. Relative gene expression was calculated using the 2^–ΔΔ*Ct*^ method (Zhang F. et al., 2020).

### Statistical Analysis

Statistical analyses were performed using SPSS 21.0 software (SPSS Inc., Chicago, IL, United States). All RNA data were expressed as the median level. For comparisons between more than two groups, the Kruskal-Wallis test was used. *P*-values < 0.05 were considered statistically significant. GraphPad Prism software version 8 (GraphPad Software, La Jolla, CA, United States) was used to make boxplots, heatmap graphs and scatterplots.

The article "Abnormal Mitochondria-Endoplasmic Reticulum Communication Promotes Myocardial Infarction" was retracted in 2022. Reasons: compromised peer review; original data or images not available; unreliable data.

## Results

### Hypoxia Activates Mitochondrial Division and Oxidative Stress in Cardiomyocytes

To mimic myocardial infarction *in vitro*, we subjected cardiomyocytes to hypoxia treatment for 24 h. Then, to determine whether hypoxia induced cardiomyocyte injury by damaging mitochondria, we used an immunofluorescence assay to detect changes in mitochondrial division. Under normal conditions, cardiomyocytes exhibited a round mitochondrial morphology, and the average mitochondrial length was ∼9.8 μm (Figures 1A–C). However, when cardiomyocytes were exposed to hypoxia, the proportion of fragmented mitochondria increased, so the average mitochondrial length decreased to ∼4.3 μm.

**FIGURE 1:** Hypoxia induces mitochondrial division and oxidative stress in cardiomyocytes. **(A–C)** Cardiomyocytes were subjected to hypoxia to mimic myocardial infarction *in vitro*, and an immunofluorescence assay was used to detect the mitochondrial morphology. The average length of the mitochondria and the percentage of fragmented mitochondria were recorded. **(D–G)** qRT-PCR was used to analyze the transcription of *Drp1*, *Mff*, *Mid49*, and *Mid51* in cardiomyocytes subjected to hypoxia. **(H,I)** MtROS were detected through an immunofluorescence assay. **(J,K)** ELISAs were used to analyze anti-oxidative enzyme activity. *p < 0.05 vs. control group.

To further evaluate the activation of mitochondrial division in hypoxia-treated cardiomyocytes, we used quantitative real-time PCR (qRT-PCR) to analyze the transcription of genes involved in mitochondrial division. As shown in Figures 1D–G, *Drp1*, *Mff*, *Mid49*, and *Mid51* mRNA levels were significantly elevated in cardiomyocytes under hypoxic conditions. These data confirmed that hypoxia activated mitochondrial division in cardiomyocytes.

We also monitored mitochondrial oxidative stress under hypoxic conditions. The levels of mtROS were significantly greater in hypoxia-treated cardiomyocytes than in control cardiomyocytes (Figures 1H,I), suggesting that hypoxia treatment created an oxidative stress microenvironment. In addition, enzyme-linked immunosorbent assays (ELISAs) demonstrated that glutathione (GSH), SOD, and glutathione peroxidase (GPX) levels were markedly downregulated in hypoxia-treated cardiomyocytes (Figures 1J–K), confirming that hypoxia induced mitochondrial oxidative stress in cardiomyocytes.

### The mtROS/JNK Pathway Induces Cardiomyocyte Death

Considering that hypoxia damaged mitochondria and generated mtROS in cardiomyocytes, we wondered whether the JNK pathway (which is activated by mitochondrial damage and oxidative stress) contributed to cardiomyocyte death under hypoxic conditions. Western blotting illustrated that the JNK pathway was activated in hypoxia-treated cardiomyocytes compared with control cells (Figures 2A,B). Interestingly, the application of mitoQ, a neutralizer of mtROS, prevented JNK activation in hypoxia-treated cardiomyocytes, suggesting that mtROS were upstream inducers of the JNK pathway. Accordingly, an immunofluorescence assay indicated that hypoxia elevated JNK expression in cardiomyocytes, whereas mitoQ prevented this alteration (Figures 2C,D).

The article "Abnormal Mitochondria-Endoplasmic Reticulum Communication Promotes Myocardial Infarction" was retracted in 2022. Reasons: compromised peer review; original data or images not available; unreliable data.

**FIGURE 2:** The mtROS/JNK pathway induces cardiomyocyte death. **(A,B)** Western blotting was used to analyze phosphorylated JNK levels in cardiomyocytes subjected to hypoxia. The mtROS neutralizer mitoQ was used to attenuate mtROS levels in cardiomyocytes. **(C,D)** An immunofluorescence assay was used to detect phosphorylated JNK levels in cardiomyocytes subjected to hypoxia. **(E)** Cardiomyocyte viability was measured using a CCK-8 assay. **(F)** An ELISA was used to analyze caspase-3 activity in cardiomyocytes subjected to hypoxia or treated with mitoQ. *p < 0.05 vs. control group.

To assess whether cardiomyocyte death was under the control of the mtROS/JNK pathway, we employed a Cell Counting Kit 8 (CCK-8) assay to analyze cardiomyocyte viability. As shown in Figure 2E, hypoxia reduced cardiomyocyte viability, while mitoQ inhibited this effect. Moreover, an ELISA demonstrated that hypoxia promoted caspase-3 activity in cardiomyocytes, whereas mitoQ significantly suppressed it (Figure 2F). These results illustrated that the mtROS/JNK pathway induced cardiomyocyte death under hypoxic conditions.

### Fis1 and BAP31 Are Upregulated in Cardiomyocytes Under Hypoxic Conditions

Previous studies have demonstrated that Fis1 and BAP31 promote mitochondrial division in the infarcted heart; thus, we analyzed Fis1 and BAP31 expression in cardiomyocytes exposed to hypoxia. In a qRT-PCR assay, *Fis1* and *BAP31* mRNA levels increased rapidly in hypoxia-treated cardiomyocytes (Figures 3A,B). Likewise, Western blotting revealed that hypoxia induced Fis1 and BAP31 protein expression in cardiomyocytes (Figures 3C–E).

**FIGURE 3:** Hypoxia induces Fis1 and BAP31 expression in cardiomyocytes. **(A,B)** qRT-PCR was used to analyze *Fis1* and *BAP31* mRNA levels in cardiomyocytes subjected to hypoxia or treated with mitoQ. **(C–E)** Western blotting was used to detect Fis1 and BAP31 expression in cardiomyocytes subjected to hypoxia or treated with mitoQ. *p < 0.05 vs. control group.

### Silencing of *Fis1* or *BAP31* Attenuates Mitochondrial Division and Mitochondrial Oxidative Stress

To determine whether Fis1 and BAP31 contributed to mitochondrial damage in cardiomyocytes exposed to hypoxia, we transfected cardiomyocytes with small interfering RNAs (siRNAs) against *Fis1* or *BAP31*. Then, we assessed mitochondrial division and mitochondrial oxidative stress under hypoxic conditions. As shown in Figures 4A–C, silencing of *Fis1* or *BAP31* increased the number of round mitochondria in cardiomyocytes under hypoxic conditions. In addition, the average length of mitochondria in hypoxia-exposed cardiomyocytes increased to ∼8.7 μm upon the silencing of *Fis1* or *BAP31*. These data indicated that silencing *Fis1* or *BAP31* could inhibit or attenuate mitochondrial division.

The article "Abnormal Mitochondria-Endoplasmic Reticulum Communication Promotes Myocardial Infarction" was retracted in 2022. Reasons: compromised peer review; original data or images not available; unreliable data.

**FIGURE 4:** Silencing of *Fis1* or *BAP31* attenuates mitochondrial division and oxidative stress. **(A–C)** Cardiomyocytes were subjected to hypoxia to mimic myocardial infarction *in vitro*. SiRNAs were used to attenuate *Fis1* or *BAP31* expression in cardiomyocytes. Then, an immunofluorescence assay was used to detect the mitochondrial morphology. The average length of the mitochondria and the percentage of fragmented mitochondria were recorded. **(D,E)** MtROS were detected using an immunofluorescence assay. **(F,G)** ELISAs were used to analyze anti-oxidative enzyme activity. *p < 0.05.

Next, we analyzed whether Fis1 and BAP31 promoted mitochondrial oxidative stress in cardiomyocytes under hypoxic conditions. Silencing of *Fis1* or *BAP31* significantly suppressed mtROS production in hypoxia-treated cardiomyocytes (Figures 4D,E). Moreover, anti-oxidative enzyme activity in hypoxic cardiomyocytes increased in response to *Fis1* or *BAP31* silencing (Figures 4F–G). These results suggested that the inhibition of *Fis1*/*BAP31* could normalize mitochondrial redox biology in cardiomyocytes.

### Inhibition of *Fis1*/*BAP31* Prevents JNK Activation and Promotes Cardiomyocyte Survival

Considering that Fis1 and BAP31 induced mitochondrial division and oxidative stress, we wondered whether these proteins also stimulated the JNK pathway and mitochondria-dependent cell death in cardiomyocytes. Western blotting demonstrated that hypoxia increased JNK phosphorylation in cardiomyocytes, whereas siRNAs against *Fis1* or *BAP31* suppressed this alteration (Figures 5A,B). An ELISA measuring JNK activity also illustrated that the loss of *Fis1*/*BAP31* reduced JNK activation in hypoxia-exposed cardiomyocytes (Figure 5C).

**FIGURE 5:** Inhibition of *Fis1*/*BAP31* prevents JNK activation and promotes cardiomyocyte survival. **(A,B)** Cardiomyocytes were subjected to hypoxia to mimic myocardial infarction *in vitro*. SiRNAs were used to attenuate *Fis1* or *BAP31* expression in cardiomyocytes. Then, Western blotting was used to analyze phosphorylated JNK levels in cardiomyocytes subjected to hypoxia. **(C)** An ELISA was used to detect JNK activity. **(D)** A CCK-8 assay was used to analyze the viability of cardiomyocytes. **(E,F)** The number of TUNEL-positive cells was measured using immunofluorescence. *p < 0.05.

The article "Abnormal Mitochondria-Endoplasmic Reticulum Communication Promotes Myocardial Infarction" was retracted in 2022. Reasons: compromised peer review; original data or images not available; unreliable data.

To understand the influence of Fis1/BAP31 on cardiomyocyte death, we conducted a CCK-8 assay. As shown in Figure 5C, hypoxia reduced cardiomyocyte viability, whereas this effect was not evident in cardiomyocytes transfected with siRNAs against *Fis1* or *BAP31*. To quantify the number of apoptotic cardiomyocytes, we performed terminal deoxynucleotidyl transferase dUTP nick end labeling (TUNEL) staining (Figures 5D,E). The percentage of apoptotic cardiomyocytes was ∼5% under normal conditions, and increased significantly in response to hypoxia. However, loss of *Fis1* or *BAP31* reduced the percentage of apoptotic cardiomyocytes to ∼8% (Figures 5E,F). These data confirmed that the inhibition of *Fis1*/*BAP31* prevented JNK activation and promoted cardiomyocyte survival under hypoxic conditions.

## Discussion

Myocardial infarction is characterized by cardiomyocyte death, but the mechanisms are not fully understood, despite basic and clinical research efforts (Bacmeister et al., 2019; Hofbauer et al., 2019; Behrouzi et al., 2020; Golforoush et al., 2020). In the present study, we found that mitochondrial oxidative stress-induced JNK activation may be the upstream trigger of cardiomyocyte death under hypoxic conditions. The inhibition of mitochondrial oxidative stress prevented hypoxia-induced JNK activation and thus enhanced the resistance of cardiomyocytes to hypoxic stress.

The results of this study are in accordance with previous findings. For example, inhibiting the JNK pathway using sesamin was found to reduce cardiomyocyte apoptosis and inflammation in a rat model of myocardial infarction (Fan et al., 2017). In contrast, overexpression of tumor necrosis factor (TNF) receptor-associated factor 1 was reported to activate the JNK pathway and therefore aggravate myocardial ischemia/reperfusion injury (Xu et al., 2019). Molecular experiments have indicated that the inhibition of the JNK pathway reduces the rate of mitochondrial permeability transition pore opening (Li et al., 2016), although mitochondrial oxidative stress has been regarded as the upstream inducer of JNK. Interestingly, suppression of the JNK pathway was found to attenuate mtROS production in a model of post-infarction cardiac remodeling (Yang et al., 2018), so it is an open question whether mitochondrial oxidative stress and JNK exert positive feedback on each other. In the present study, we observed that mtROS induced the JNK pathway in cardiomyocytes under hypoxic conditions.

The article "Abnormal Mitochondria-Endoplasmic Reticulum Communication Promotes Myocardial Infarction" was retracted in 2022. Reasons: compromised peer review; original data or images not available; unreliable data.

Mitochondrial division morphologically alters mitochondria to elevate the number of these organelles in response to different stimuli (Akbari et al., 2019; Wang et al., 2019; Shanmughapriya et al., 2020; Zhou and Tan, 2020). Increasing the population of mitochondria enhances the ATP production efficiency under physiological conditions (Currais, 2015; Bai et al., 2020; Makrecka-Kuka et al., 2020). Therefore, although cardiomyocytes have a limited capacity to proliferate, they can employ mitochondrial division to accelerate their metabolic rate. Unfortunately, pathological mitochondrial fission harms heart tissue by promoting the uneven distribution of mitochondrial DNA into the mitochondrial offspring (Del Campo, 2019; Li et al., 2019; Burtscher, 2020). Damaged mitochondrial DNA cannot sufficiently generate the mitochondrial respiratory complexes, so ATP production is suppressed in cardiomyocytes with abnormal mitochondrial fission.

A previous report indicated that inhibiting mitochondrial fission markedly reduced post-infarction cardiac injury by improving the mitochondrial performance (Liu et al., 2019). Moreover, mitochondrial calcium uniporter overexpression was shown to induce myocardial ischemia/reperfusion by activating mitochondrial fission (Guan et al., 2019). In the present study, mitochondrial division was found to be the upstream inducer of mtROS overproduction and JNK pathway activation in cardiomyocytes exposed to hypoxia. Interestingly, recent studies have indicated that mitochondrial fission is also induced by JNK; for example, knocking out Macrophage stimulating 1 was reported to inhibit mitochondrial fission by preventing JNK activation in myocardial infarction (Wang and Song, 2018; Depoix et al., 2020). This seems to be an injury amplification mechanism that promotes cardiomyocyte death (Zhou et al., 2021; Zhu et al., 2021).

The novel finding of this study is that mitochondrial division is highly dependent on ER-mitochondria contact. BAP31 is an ER protein that regulates intracellular calcium homeostasis and ER stress (Zhang J. et al., 2020). Fis1 is a mitochondrial protein that functions with Drp1 to promote mitochondrial division. Interestingly, we have provided ample evidence that Fis1 and BAP31 induce not only mitochondrial division, but also mitochondrial damage. Loss of *BAP31* or *Fis1* reduced mitochondrial oxidative stress and increased cardiomyocyte survival under hypoxic conditions, suggesting that the cooperation between BAP31 and Fis1 promotes mitochondrial division and determines cardiomyocyte fate. Considering the localization of BAP31 and Fis1, communication between mitochondria and the ER may help to initiate mitochondrial division. This concept has been proposed by other researchers, but it has not been validated in cardiovascular disorders. Our findings suggested that mitochondria-ER communication induces abnormal mitochondrial division and cardiomyocyte death during myocardial infarction.

The article "Abnormal Mitochondria-Endoplasmic Reticulum Communication Promotes Myocardial Infarction" was retracted in 2022. Reasons: compromised peer review; original data or images not available; unreliable data.

Overall, our results illustrated that cardiomyocyte death during myocardial infarction is caused by mtROS overload and subsequent JNK activation. Cooperation between mitochondria and the ER promotes mitochondrial division, the initial inducer of mitochondrial oxidative stress in cardiomyocytes. However, there are several limitations to the present study. First, animal experiments are necessary to verify our *in vitro* findings. Second, the molecular mechanism whereby BAP31 interacts with Fis1 remains unclear. Third, a treatment approach specifically inhibiting mitochondria-ER contact or BAP31/Fis1 binding is lacking. Additional research is needed to develop such an inhibitor.

## Data Availability Statement

The original contributions presented in the study are included in the article/supplementary material, further inquiries can be directed to the corresponding author/s.

## Author Contributions

DC, CL, and JZ conceived the study and wrote the manuscript. FH and WL performed the experiments and contributed the data. All authors have approved the final version of the manuscript.

## Conflict of Interest

The authors declare that the research was conducted in the absence of any commercial or financial relationships that could be construed as a potential conflict of interest.

## Publisher’s Note

All claims expressed in this article are solely those of the authors and do not necessarily represent those of their affiliated organizations, or those of the publisher, the editors and the reviewers. Any product that may be evaluated in this article, or claim that may be made by its manufacturer, is not guaranteed or endorsed by the publisher.
